# Serotonin 5-HT_7_ receptor agonist, LP-211, exacerbates Na^+^, K^+^-ATPase/Mg^2+^-ATPase imbalances in spinal cord-injured male rats

**DOI:** 10.1186/s13000-015-0397-7

**Published:** 2015-09-14

**Authors:** Abbas Norouzi-Javidan, Javad Javanbakht, Fardin Barati, Nahid Fakhraei, Fatemeh Mohammadi, Ahmad Reza Dehpour

**Affiliations:** Brain and Spinal Cord Injury Research Center, Neuroscience Institute, Tehran University of Medical Sciences, Tehran, Iran; Experimental Medicine Research Center, School of Medicine, Tehran University of Medical Sciences, Tehran, Iran; Department of Pharmacology, School of Medicine, Tehran University of Medical Sciences, P.O. Box 13145-784, Tehran, Iran

## Abstract

**Background:**

The observed controversy that N-(4-cyanophenylmethyl)-4-(2-diphenyl)-1-piperazinehexanamide (LP-211), a selective serotonin (5-HT_7_) receptor agonist, may either modify or exacerbate imbalances in serum electrolyte concentrations and renal tissue of spinal cord trauma cases has not been reported yet. The aim of this study was to better understand the effects of a new 5-HT_7_ receptor agonist, LP-211, on serum electrolyte changes in spinal cord injured- (SCI) rats.

**Methods:**

Sixty male rats were assigned to the following groups: A) Intact (saline as vehicle, 1 ml/kg, i.p.), B) Intact [LP-211, (0.003–0.3 mg/kg, i.p.)], C) Sham-operated [laminectomy + vehicle (1 ml/kg, i.p.)], D) Sham-operated [laminectomy + LP-211 (0.003–0.3 mg/kg, i.p.)], E) Treatment [laminectomy + spinal trauma (SCI) + vehicle (1 ml/kg, i.p.)], F) Treatment [laminectomy + spinal trauma + LP-211 (0.003–0.3 mg/kg, i.p.)]. SCI was performed by placing an aneurysm clip, extradurally at the level of T10. After two weeks, LP-211 was administered cumulatively and each dose was injected (i.p.) with 20 min interval. At the end of the experiment, blood samples were collected for biochemical evaluations of the electrolytes employing standard commercial kits.

**Results:**

The present results indicate elevated serum levels of Na^+^, K^+^, and Mg^2+^ in SCI rats and significant differences demonstrated between the groups [*P* < 0.001, F(5, 35) = 23.92], [*P* < 0.001, F(5, 35) = 67.63], [*P* < 0.001, F(5, 35) = 71.144], respectively. So that, in groups B, D and F, there was a significant increase in K^+^ and Mg^2+^ serum levels compared to the groups A, C, and E (*P* < 0.001). Furthermore, Na^+^ serum levels in SCI (LP-211), laminectomy (LP-211), and intact (LP-211) groups tended to be statistically lower than SCI (saline), laminectomy (saline) and intact (saline) groups. Infact, hyponatremia, hyperkalemia and hypermagnesemia was obtained in group F. Nevertheless, in the remaining measured serum electrolytes such as calcium (Ca^2+^), iron (Fe^2+^) and phosphorus (P^3−^), chlorine (Cl^−^), copper (Cu^+^), and zinc (Zu^+^), no significant changes were observed.

**Conclusion:**

It was shown that acute additive LP-211 treatments in the SCI group led to hyponatremia, hyperkalemia and hypermagnesemia, it may be stated that LP-211 treatment as a promising candidate for treating SCI complications in some systems especially urinary tract might take into consideration and further studies would be needed to clarify its benefits or drawbacks. The observed discrepancies, nevertheless; will also pose new questions. Altogether, this will ultimately contribute to further understanding the pathophysiological role regarding 5-HT_7_ receptor activation.

## Background

Traumatic spinal cord injury (SCI) is a major clinical problem with permanent neurological deficits and a broad range of secondary complications [1]. The pathophysiology of acute SCI involving primary and secondary mechanisms of injury is highly complex and not clearly understood. Primary events occur at the time of trauma and related to mechanical damage and after primary injury, further pathophysiological processes such as hypoxia, edema and inflammation, altered blood flow and changes in microvascular permeability are triggered; thus, lesions greatly enlarge and worsen by secondary injury [2, 3]. Secondary events develop hours to days after trauma, which includes a cascade of biochemical and cellular processes, such as electrolyte abnormalities, formation free radicals, vascular ischemia, edema, posttraumatic inflammatory reaction together with demyelination and further cell death by necrotic and apoptotic pathways [4–6]. In parallel, several studies have revealed that one consequence of trauma to the spinal cord is an increase in lipid peroxidation and a decrease in the activity of the critical membrane-bound enzymes such as Na^+^-K^+^-activated ATPase and Na^+^-K^+^/Mg^+2^ ATPase [7–10].

Nowadays, much attention has been focused on the biochemical changes of secondary injury in spinal cord trauma. In parallel to, the degree of exchange of Na^+^, K^+^ and Mg^2+^ between tissues and plasma varies greatly. So that, most studies have shown changes in intracellular Mg^2+^ concentration over the physiologic-pathophysiologic range would significantly affect K^+^ secretion. Furthermore, in SCI intracellular effects of Mg-ions are opposite to Ca-ions in competition at K-ion channels, in Na^+^-K^+^/Mg^+2^ ATPase activity, cAMP/cGMP concentration and Ca-ion currents in pre- and postsynaptic membranes [11, 12]. To support this idea, multiple studies have demonstrated that traumatic spinal injury causes a decrease in intracellular free potassium and magnesium concentrations, which correlated with injury severity, and is associated with a decrease in total tissue K^+^ and Mg^2+^concentrations [13–16].

The 5-HT_7_ receptor was the last member of the 5-HT receptor family to be identified and was cloned independently by three laboratories in 1993 [17, 18]. These primary studies demonstrated that the 5-HT_7_ receptor is positively coupled to adenylate cyclase through the stimulatory Gs protein, with a pharmacological profile distinct from that of all other 5-HT receptors [19]. Pharmacological and genetic tools targeting the 5-HT_7_ receptor in animal models have implicated this receptor in various pathophysiological processes, including: regulation of body temperature [20], circadian rhythms [21], learning and memory [22]. Inflammatory processes in the CNS [23], smooth muscle relaxation of cerebral arteries [24], mood disorders [25, 26], and pain [27].

The Na^+^-K^+^ pump is a ubiquitous membrane protein that catalyzes the active transport of K^+^ into cells and Na^+^ out of cells against their electrochemical gradient. Na^+^-K^+^ pump activity is regulated by a variety of hormones, neurotransmitters, and growth factors. 5-HT, in particular, activates the Na^+^-K^+^ pump in the brain [28], kidney [29], and vascular smooth muscle [30]. Indeed, stimulation of the Na^+^-K^+^ pump by 5-HT has been proposed to mediate the inhibitory effect that 5-HT exerts on vascular smooth muscle tone [31–33]. The cellular mechanism for 5-HT-induced contraction of airway smooth muscle has been well characterized and is similar to that of other contractile receptor agonists. 5-HT interacts with specific receptors to stimulate inositol phosphate metabolism, Ca^2+^ mobilization, and protein kinase C activation [34–38]. In contrast, the mechanism of relaxes vascular smooth muscle by 5-HT via 5-HT_7_ receptors is unknown.

In recent years, considerable efforts have been focused on the development of selective 5-HT_7_ receptor agonists and antagonists [39, 40]. Although the effects of selective 5-HT_7_ agonism/antagonism have been studied in several animal models where it has been shown to have anxiolytic [41–43], antidepressant [44–46], antipsychotic-like hyponatremia, hyperkalemia and hypermagnesemia in [47, 48] and anti-inflammatory effects [49], to our knowledge, no current data are available on the effects of 5-HT_7_ receptor agonists/antagonists in serum electrolyte concentrations. Among these, the 5-HT_7_ receptor subtype is the target of LP-211, a newly synthesized selective agonist [50–52]. Therefore, in this manuscript, for the first time, we attempt to investigate low-term effects of LP-211, on serum electrolyte profile, using rat model of SCI.

## Methods

### Animals

All experimental protocols were approved by the local animal care committee in accordance with Tehran University of Medical Sciences guidelines for the care and use of laboratory animals. In the current study, 60 adult male Wistar albino rats (Pasteur Institute, Tehran, Iran), weighing 300–350 g with 7–8 weeks old were utilized. The animals were kept in individual propylene cages under standard laboratory conditions. Rats were maintained on a 12 h light/dark cycle at 23 ± 2 °C and 50 ± 5 % humidity. The animals were kept in standard room conditions and fed with standard rat diet and water ad libitum.

### Chemicals

LP-211(N-(4-cyanophenylmethyl)-4-(2-diphenyl)-1-piperazinehexanamide (SERVA Chemical Co., New York) was dissolved in distilled water.

### Treatment

Successive doses (0.003–0.3 mg/kg, i.p.) were administered cumulatively at short intervals (20 min maximum). The drugs doses were in accordance with dosages determined in previous studies [52–54]. All drug solutions were administered in a volume of 0.5 ml.

### Laminectomy procedures

All surgery was carried out in sterilized condition. Animals were anesthetized by intraperitoneal injection of a mixture of ketamine hydrochloride (75 mg/kg) and xylazine hydrochloride (5 mg/kg). Their dorsal regions were shaved and cleaned with povidone Iodine 10 %. Under the sterile technique, after a dorsomedial incision on skin, a laminectomy was performed between vertebral levels T9–T11 to expose the underlying T10 spinal cord, and the spinal cord was exposed microsurgically [9]. After the incision of the dermal and sub-dermal tissues at the midline, paravertebral muscles were dissected bluntly exposing the lamina bilaterally. Complete laminectomies were performed, exposing the spinal cord at T9–T11. Strict bleeding control was performed using bone wax and bipolar coagulator. The crushing or SCI was produced by using the aneurysm clips (Yasargil FE 760) for 1 min with a closing force of 180 g on the spinal cord at room temperature in T10 level [52, 53]. After carefully removing the aneurysm clip, the fascia and the skin were sutured separately using silk stitches. For the sham-operated-operation, only the skin and muscles in the thoracic vertebral level were removed but the dura was kept intact. Following surgery and or/upon SCI, animals received antibiotics enrofloxacin 2.5 % intramuscular in the dose of 2.5 ml/Kg of body weight for three days. Until termination of the experiment the welfare of the rats was routinely checked. Furthermore, biochemical analysis for the electrolytes ions was performed 14 days after SCI.

### Experimental groups

The rats were randomly divided into six groups of ten as follows:

1. Intact (saline as vehicle): No SCI or treatment was performed. Samples were obtained to determine baseline biochemical values.
2. Intact (LP-211): No SCI or treatment was performed: samples were obtained to determine baseline biochemical values.
3. Sham-operated (laminectomy + vehicle): rats underwent only a simple laminectomy. No SCI or treatment was performed.
4. Sham-operated (laminectomy + LP-211): rats underwent a simple laminectomy and treatment. No SCI was performed.
5. Treatment (laminectomy + spinal trauma + vehicle): Laminectomy and trauma was performed. Rats received vehicle immediately following SCI.
6. Treatment (laminectomy + spinal trauma + LP-211): Laminectomy and trauma was performed. Drugs were diluted with sterile saline and given intraperitoneally (i.p.).

### Assessment of biochemical analysis

All animals were anesthetized (ketamine hydrochloride 10 % + xylazine 2 %, in 80 and 5 mg/kg doses, respectively). Blood samples were collected by cardiac puncture. After this procedure, animals were sacrificed under ketamine–xylazine (KX) anesthesia.

For biochemical analyses, of blood was collected (5 ml), in order to obtain serum samples. Serum was prepared from whole blood without any anticoagulant. Plasma was prepared from heparinized blood, separated by centrifugation at 1650 g for 10 min and stored at 4 °C for later use (MSE Minor, England). Serum samples were separated into the sterile plain tubes and stored in the refrigerator for future analyses. All the analyses were completed within 48 h of the sample collection.

### Serum electrolytes

Serum levels of Magnesium (Mg^2+^), Calcium (Ca^2+^), Iron (Fe^2+^) and Phosphorus(P^3−^) were determined with the aid of commercial kits from Wiener Lab and the BT 3000 Plus Analyzer. Sodium (Na^+^), Chlorine (Cl^−^), Potassium (K^+^), Copper (Cu^+^), and Zinc (Zu^+^) levels were determined using a Flame Photometer and analytical standard ion solutions. The samples were diluted 100 × in Milli Q water.

### Statistical analysis

The analyses were performed using SPSS (v. 18). The results are given as means ± SE. Differences between groups were assessed using a one-way analysis of variance (ANOVA) and followed by Tukey post test. The values of *P* < 0.05, was considered statistically significant.

## Results

The serum levels of Na^+^, K^+^ and Mg^2+^ are summarized in Figs. 1, 2 and 3.

**Fig. 1:** Histogram comparing the effects of saline (vehicle) and LP-211 on serum sodium levels in rats. The data is expressed as mean ± standard deviation (SD). Significantly different from intact ^###^(*p* < 0.001). Significantly different from laminectomy and SCI ***(*p*< 0.001). Statistical analysis was performed by oneway ANOVA and Tukey post-hoc tests

**Fig. 2:** Histogram comparing the effects of saline (vehicle) and LP-211 on potassium levels in rats. The data is expressed as mean ± standard deviation (SD). Significantly different from intact ^###^(*p* < 0.001). Significantly different from laminectomy and SCI **(*p* < 0.01), ***(*p* < 0.001). Statistical analysis was performed by oneway ANOVA and Tukey post-hoc tests

**Fig. 3:** Histogram comparing the effects of saline (vehicle) and LP-211 on magnesium levels in rats. The data is expressed as mean ± standard deviation (SD). Significantly different from intact ^###^(*p* < 0.001).Significantly different from laminectomy and SCI ** (*p* < 0.01), ***(*p* < 0.001). Furthermore, serum magnesium levels measured in the SCI (Saline) group was significantly higher than levels measured in laminectomy (Saline) rats *(*p* < 0.05). Statistical analysis was performed by one-way ANOVA and Tukey post-hoc tests

The Na^+^ levels were significantly higher in the intact (saline) group compared with intact (LP-211) group (*p* < 0.001), SCI (saline), laminectomy (saline), laminectomy (LP-211) and SCI (LP-211) groups (*p* < 0.001). Furthermore, the serum levels of Na^+^ in SCI (LP-211), laminectomy (LP-211),and intact (LP-211) groups tended to be lower than SCI (saline), laminectomy (saline) and intact (saline) groups, respectively, the difference was statistically significance (*P* < 0.001). In addition, serum Na^+^ levels in the non-treatment groups (e.g. intact and sham-operated) tended to be higher than in the treatment groups, the difference was significant (*P* < 0.001). Serum Na+ levels did significant differences compared between the different groups. Additionally, the administration of LP-211 significantly reduced the serum Na+ levels compared with the trauma, sham-operated, and intact groups (*P* < 0.001) (Fig. 1).

K+ levels in the serum were found to be significantly higher in the group SCI (LP-211), than the groups intact, sham-operated, and SCI (saline) (*p* < 0.001). So that, in the groups SCI (LP2-11) and intact (LP-211), there was a significant increase in K+ levels of the serum when compared to the groups SCI (saline) and intact (saline), respectively. Moreover, in the group SCI (saline), activities of the potassium levels were found to be significantly lower than in the group laminectomy (LP-211) (*p* < 0.01). The differences were statistically very significant not only between the groups SCI (LP-211) and laminectomy (saline), but also between the groups intact (saline) and intact (LP-211) (*p* < 0.001). Therefore, treatment with LP-211 significantly prevented the reduction of k+ levels in the serum. On the other hand, LP-211 administration significantly augmented the raises in the serum k+ levels, with respect to control (Fig. 2).

On the other hand, serum Mg^2+^ levels were found to be significantly increased in the trauma group when compared with both the control and the sham-operated groups (*P* < 0.001 for both). Nevertheless, Mg^2+^ level was significantly higher in the SCI (LP-211) group than in the intact and laminectomy groups (*p* < 0.001). And also, it was significantly higher in SCI (saline) group than in laminectomy (saline) group (*p* <0.05). It was also significantly higher in the in laminectomy (LP-211) group than in the SCI (saline) group (*p* < 0.01). Taken together, they significantly decreased in the intact (saline), laminectomy (saline) and intact (LP-211) groups compared to the SCI (LP-211) group (*p* < 0.001), respectively. Explicitly, there was a significant difference in serum Mg^2+^ between the groups (*P* < 0.001) (Fig. 3). Finally, no significant changes were found in the remaining determined electrolytes.

## Discussion

This article emphasizes the major changes resulting from alterations in plasma concentrations of sodium, potassium, and magnesium after SCI. Moreover, we showed for the first time that activating 5-HT_7_ receptor by the 5-HT_7_ receptor agonist, LP-211, in experimental model of SCI, exacerbates the metabolite imbalances and elevated some serum electrolyte concentrations. We observed significantly augmented severity of serum electrolyte panel such as K^+^ and Mg^+2^ in rats that received treatment. In our study, hypermagnesemia and hyperkalemia were observed after spinal injury and LP-211 enhances these changes.

We have determined the serum Mg^2+^ concentration and demonstrate that following traumatic injury, serum Mg^2+^ concentration increases and Mg^2+^ could affect a number of factors thought to be involved in the secondary injury processes, including oxidative phosphorylation [55], activity of excitatory amino acids [56], opiate receptors [57], and eicosanoid synthesis [55]. Nevertheless, the post-traumatic decline in Mg^2+^ may be a critical early factor in the development of irreversible tissue damage following SCI. Moreover, in agreement with our data, several studies demonstrated that changes in potassium are linked to the observed decrease/increase in both total and free Mg^2+^ level. An association between changes in K^+^ and Mg^2+^ has long been recognized, and has been described in detail [58, 59], and these the present study showed a hypermagnesemia and hyperkalemia after spinal injury.

Consistent with our study, spinal cord injury in rats causes decreases in total tissue levels of Mg^2+^ and increase in serum Mg^2+^ [60]. Similar to those described by Vink et al., 1987 [61], it has found that traumatic SCI caused a significant increase in extracellular free- Mg^2+^ concentration, and the decline in intracellular and it is highly correlated to the severity of injury [62] and these changes of Mg^2+^ may contribute to secondary tissue damage [63].

In conducted studies by Anderson et al. [64–66] reported that laminectomy reduces spinal cord blood flow, and Na^+^-K^+^/Mg^2+^ ATPase activity. Therefore, the hypermagnesemia and hyperkalemia levels in our study and are in a good agreement.

Interactions between agonist and antagonist of 5-HT7 receptor, and their combined effects on neuronal function, have not been reported to the same extent as those effects mediated by the actions of SCI on serotonergic pathways. Nevertheless, recent studies with different receptors of 5-HT has been shown to inhibit Na^+^/K^+^-ATPase function; both indirectly, by phosphorylation of the pump via 5-HT_2c_ receptor activation in the choroid plexus of the rat [67], and directly, after addition to isolated Na^+^/K^+^-ATPase pump protein from the pig kidney [68]. This premise was also supported by the results of the present study. Moreover, studies have shown high expression of 5-HT_7_ receptor transcripts in pig cerebral blood vessels [69, 70], canine cerebral blood vessels [71, 72], rat cerebral blood vessels [73–75], and several human meningeal tissues, including the internal carotid and middle meningeal artery and smooth muscles [76].

Acute LP-211 exposure at 0.3 mmol/L, did significantly alter serum sodium, potassium and magnesium concentrations and the remaining doses did not significantly demonstrate decreased Na^+^-K^+^/Mg^2+^ ATPase pump activity compared with the high doses. This may reflect the fact that several steps contribute to regulation of the Na^+^-K^+^/Mg^2+^ ATPase pump, from 5-HT reuptake inhibition by LP-211 to 5-HT_7_ receptor activation and involvement of multiple potential signal transduction pathways. The LP-211-associated reduction in Na^+^/K^+^-ATPase function may be caused by several factors, including a decrease in the total number of Na^+^-K^+^/Mg^2+^ ATPase pump molecules and/or covalent modifications that affect pump function. Therefore, translational or post-translational changes, including covalent modifications of the Na^+^/K^+^-ATPase pump, also may contribute to diminished pump function. Phosphorylation via activation of specific 5-HT receptors is one likely possibility [67]. The consequences, after short-term LP-211 treatment, of reduced Na^+^/K^+^-ATPase activity on neuronal function need to be examined. LP-211 may lead to increased intracellular Na+ and extracellular K^+^/Mg^2+^ concentrations after acute exposure because of a decrease and increase in removal of cytosolic Na^+^ and K^+^/Mg^2+^ by the Na^+^/K^+^-ATPase pump, respectively. However, it is also possible that the decrease in Na^+^/K^+^-ATPase pump function is a compensatory response to a reduced intracellular Na^+^ and enhanced extracellular K^+^/Mg^2+^ concentrations arising from another effect of short-term drug treatment. Measurement of the electrolytes content should help to support either of these hypotheses. This reduction in Na^+^/K^+^-ATPase function almost certainly will affect cellular physiology. Experiments are now in progress to determine the significance of these changes that occur after short -term LP-211 treatment.

On the other hand, other investigations have shown that serotonin plays important roles in various microvascular responses after trauma to the cord including increase and disturbances of microvascular permeability, edema formation and reduction of blood flow [77–79]. Therefore it seems likely that the elevation of 5HT_7_ receptor accumulation in the traumatized cord in treated animals with LP-211 may partly be responsible for some of the harmful effects of the drug. Furthermore, multiple studies have proposed that 5-HT contributes to the posttraumatic decline of blood flow and edema seen in injured spinal cords [80–83].

## Conclusions

In summary, the data presented in this study show that serum k^+^ and Mg^2+^ levels were increased by LP-211, and the serum k+ and Mg^2+^ levels were higher in the LP-211 group compared with SCI with saline and sham-operated groups (*P* < 0.001), and also, the serum Na+ levels were lower in the LP-211 group compared with mentioned groups. We have hypothesized that this effect is induced the inhibition of Na^+^-K^+^/Mg^2+^ ATPase activity by the increase in lipid peroxidation levels by SCI and LP-211. The results of our study provided the first experimental evidence of the serum biochemical events of LP-211 in traumatic SCI. Therefore, in light of these results, we believe that LP-211 may not be a potential electroprotective agent for clinical trials of SCI.

To the best of our knowledge, the present study showing the negative correlation between serum electrolyte changes, SCI and LP-211 findings at comparison between groups, but future studies will be needed to reveal important explanations for the questions about the details of LP-211 mechanisms in secondary injury after spinal cord trauma on Na^+^- K^+^/Mg^2+^ ATPase activity and in order to verify this correlation in detail.

Regarding the above information, it was shown that even acute additive LP-211 treatments in the SCI group led to hyponatremia, hyperkalemia and hypermagnesemia, it may be stated that LP-211 treatment as a promising candidate for treating SCI complications in some body systems especially urinary tract might take into consideration and further studies would be needed to clarify its dose-dependent benefits or drawbacks and in SCI patients. The observed discrepancies, nevertheless; will also pose new questions. Altogether, this will ultimately contribute to the further understanding of the pathophysiological role due to 5-HT_7_ receptor activation.
